# Cost Estimates of Postnatal Care in Public Primary Care Facilities in Negeri Sembilan, Malaysia

**DOI:** 10.21315/mjms2022.29.5.10

**Published:** 2022-10-28

**Authors:** Farhana Aminuddin, Mohd Shahri Bahari, Mohd Shaiful Jefri Mohd Nor Sham Kunusagaran, Nur Amalina Zaimi, Mohd Ridzwan Shahari, Nor Zam Azihan Mohd Hassan

**Affiliations:** 1 Centre of Health Economics Research, Institute for Health Systems Research, National Institutes of Health Malaysia, Setia Alam, Selangor, Malaysia; 2 Medical Development Division, Ministry of Health Malaysia, Complex E, Federal Government Administrative Centre, Putrajaya, Malaysia

**Keywords:** postnatal care, postnatal cost, public primary care, resource allocation

## Abstract

**Background:**

Postnatal care (PNC) in Malaysia is believed to have played a role in reducing maternal and child mortality. A pilot study was thereby conducted to estimate the cost of PNC in public primary care facilities in Negeri Sembilan from the perspective of healthcare providers.

**Methods:**

This study employed a cross-sectional design that involved six public primary care facilities in Negeri Sembilan, Malaysia. The PNC-related costs data were collected between May and July 2017, utilising cost data for the year 2016 and involving 287 eligible mothers. The PNC costs were calculated using mixed top-down and activity-based costing (ABC) approaches.

**Results:**

The mean cost of PNC per patient was RM165.65 (median, RM167.12). Personnel cost was the main cost driver for PNC, which accounted for the most significant proportion of the total cost at 94.2%. Education level, type of health facilities and postnatal visits were positively associated with the total PNC cost.

**Conclusion:**

This study highlighted the average cost of PNC in the public primary care facilities in Negeri Sembilan. The cost of PNC was revealed to be primarily driven by personnel cost. The findings of this pilot study could add to the evidence base of PNC and serve as a vital reference for improving future estimates to better allocate scarce resources.

## Introduction

Global initiatives in maternal and newborn health to reduce morbidity and mortality remain a priority in the new Sustainable Development Goals agenda through 2030 (1). In 2018, about 2.5 million children died during the first month of their life (2), accounting for 47% of all child deaths under the age of five years old. Similar to antenatal care, postnatal care (PNC) is amongst the primary interventions aimed to reduce maternal and child mortality worldwide (3–5). In Malaysia, maternal and child health services have rapidly improved especially at the turn of the millennium. This achievement reflects a strategic approach, which includes improved overall access to quality healthcare, increased personnel skills to manage pregnancy and delivery complications, expanded provision of services in underserved areas, improved modern maternal health services, improved efficiency of referral and feedback systems to prevent delays and enhanced monitoring system (6).

Malaysia operates a dual-tiered healthcare system: a network of tax-funded public provider and a thriving private sector. The governmental or public healthcare sector, which is heavily subsidised through budget allocations, caters to the bulk (65%) of the population. Except for a registration fee of RM1.00 or USD0.30 per visit (7), healthcare services provided by the public primary care facilities are free of charge including maternal care. Thus, it is less likely for individuals to encounter a financial burden to receive PNC services in Malaysia.

The PNC services in Malaysia are provided at the first level of care (primary care facilities) and the referral hospital for the backup care and services. In 2013, the Ministry of Health (MOH) Malaysia released a guideline to ensure appropriate care and safe practices for postnatal mothers (8). According to this guideline, the postnatal period lasts for 42 days, from the end of labour until the genital tract returns to normal. Alternatively, the postnatal period begins just after childbirth and through the first 6 weeks, as defined by the World Health Organization (9). According to the MOH, a PNC visit by the health personnel should be carried out at least nine times after a normal delivery (scheduled at day-1, 2, 3, 4, 6, 8, 10, 15 and 20 of puerperium) with an additional visit to a healthcare practitioner at day-30. During these visits, any maternal and child health complications experienced may necessitate additional postnatal visits and appropriate referrals to a clinic or hospital.

Sustaining the current low level of maternal mortality in Malaysia and subsequently reducing it even further will require continued commitment, human resources, financial resources and innovative programme platforms. Moreover, providing the best maternal and child healthcare delivery for the citizens would require a significant allocation of expenditure (10). In 2020, around 13.6% (RM1.68 billion) of the total primary care budget (RM12.40 billion) was allocated for maternal and child health, family planning and counselling (11). However, details on the specific allocation for providing PNC is unknown. It is unfortunate because this information is important to provide evidence for policymakers concerning the cost of providing PNC services in addition to providing insights on the effectiveness of decision making.

Existing literature on the PNC cost is rather limited despite having a wide variation of studies reporting on the cost of maternal care and antenatal care. According to studies conducted on PNC, the PNC cost per visit reported in a few countries were as follows: £128.03–£182.32 in the United Kingdom (12); < ₦288 in Northern Nigeria (13); USD8.50–USD13.40 in Ethiopia (14); USD5.04 in Bangladesh (15) and USD8.30–USD17.68 in Somalia (16).

Since there is a lack of studies regarding the total cost of PNC in particular, this study becomes potentially significant. Given this is a small-scale pilot study involving only one state in Malaysia and a few primary care facilities, it can eventually serve as a preliminary basis to inform current priorities in Malaysia. Besides, this study may provide relevant estimates for policymakers to evaluate whether the resources currently available for PNC are effectively and efficiently allocated. Thus, this study aims to estimate the PNC cost in selected public primary care in Negeri Sembilan from the perspective of healthcare providers.

## Methods

### Study Site

This study was conducted in Negeri Sembilan, a state in Malaysia that lies on the western coast of Peninsular Malaysia. Negeri Sembilan was chosen due to high maternal mortality rates among other states in Malaysia. This state has seven districts with a collective population of 1.12 million as of 2018 (17). A total of 42 primary care facilities in Negeri Sembilan that provide antenatal and postnatal services to the community were listed and formed the sampling frame. A multistage stratified random sampling methodology was then employed to group the facilities into six types (Table 1) based on the daily patient attendance of the primary care facilities (18). As a result, six public primary care facilities (one from each type) were randomly selected from three district health offices as the study site for this study.

### Study Design and Sample Size Estimation

Quantitative research involving a community-based cross-sectional study was conducted among selected postnatal mothers. Data involving 287 women who had given birth between 1 January 2016 to 31 December 2016 were collected between May 2017 and July 2017 by qualified study investigators at the selected study sites. Women who delivered in the selected study sites but sought PNC services elsewhere were excluded from this study.

The sample size was determined using the open-Epi software calculator based on the proportion for one sample. With an assumption of the standard normal distribution corresponding to 95% confidence interval, an anticipated proportion of outcome variable using the birth rate for Negeri Sembilan in 2016 at 16.4%, a margin of error assumed at 1.0%, a final minimum sample size of 274 was required by adding a 20.0% dropout rate.

### Cost Data Identification, Collection and Calculation

This study was conducted from the point of view of healthcare providers, thus, the costs were calculated based on the expenditures of the providers. To estimate the costs, a step-down costing methodology combined with activity-based costing (ABC) was employed in this study. The cost data collected included the capital and recurrent costs. A capital cost is costs incurred for resources that have been used for more than a year, such as building and medical equipment. In this study, the cost of medical equipment was annualised at a discount rate of 3% over the useful lifespan of 10 years. A recurrent cost on the other hand is resources that are expected to be consumed or replaced within 1 year, such as personnel, facility utilities, laboratory tests, consumables and drugs. Details of each component in the recurrent costs included in this study are described in Table 2.

The details of the mixed step-down and ABC approach are summarised in Table 3. The step-down approach began with the total expenditure divided by the total output value (number of postnatal visits), to give an average cost per patient per year. The ABC approach allocated costs to PNC services by assigning a cost to all the items used. Data on the patient resource utilisation was collected through individual maternity record books used in the health facilities, i.e. the *Rekod Kesihatan Ibu KIK/1(b)/96 (Pindaan 2012)*, whereas data on capital costs was obtained from each health facilities records. A specially designed costing tool was developed in Microsoft Excel to allow for a systematic gathering of all required information.

### Data Analysis

Analyses were performed using the Statistical Package for the Social Sciences (SPSS) version 26 (SPSS Inc., Chicago, Illinois). Descriptive statistics were used to describe the sociodemographic profiles of the study population. A normality test was performed and confirmed that the cost data were normally distributed. For this, two-group comparisons were performed using Student’s *t*-test, while multi-group comparisons were performed using one-way ANOVA. All costs were reported in Ringgit Malaysia (RM) in the form of either mean (standard deviation [SD]) or median (interquartile range). Besides, simple and multiple linear regression analyses were performed to determine the factors associated with the outcome variable (total PNC cost). Linearity of the linear regression model was checked and satisfied using a scatter plot and normality was checked using probability (P-P) plots and histograms. The scatter plot of standardised residuals versus the predicted values showed that the model was randomly distributed. Also, the Durbin Watson statistic value (acceptable range: 1.5–2.5) was used to check the independence of errors and auto-correlations. A Durbin Watson statistic value of 1.6 for this study showed that the analysis satisfied the assumption of independence and there was no presence of auto-correlation. Variables that showed significant associations (*P* < 0.1) in the simple linear regression model were considered for the multiple linear regression analysis (19). Finally, variables that produced a *P*-value < 0.05 were considered statistically significant.

## Results

### Sociodemographic Profiles

This study involved 287 women who gave birth and utilised PNC at the selected primary care facilities in Negeri Sembilan. The sociodemographic profiles of the sample population are tabulated in Table 4. The mean age of the postnatal mothers was 29.59 (SD = 5.91) years old. The majority of the mothers were Malaysian citizens (95.8%), Malays (64.1%) and were married (95.5%). A total of 144 (50.2%) postnatal mothers had secondary school education, 75 (26.1%) had a certificate/diploma and 49 (17.1%) had a bachelor’s degree. The majority of the women were housewives (43.9%), while 36.2% were non-professional employees and 18.5% were professionals. A total of 119 women (41.5%) had uncomplicated pregnancies, whereas 168 women (58.5%) encountered problems in their pregnancy. The total PNC visit documented for all the selected women was 2,516 while the mean PNC visit recorded was around eight visits per person. The mean PNC cost according to the sociodemographic characteristics were calculated and revealed no statistical differences, except for education level and type of primary care facilities (*P* < 0.05).

Following the findings in Table 4, a linear regression analysis was run to determine the factors associated with the total PNC cost (Table 5). The education level, type of primary care facilities and the number of postnatal visits were considered in the multiple regression model (*P* < 0.05). The overall multiple regression model for the estimated total PNC cost was statistically significant, with *F*(3, 283) = 1558.73, *P* < 0.001 and *R*^2^ = 0.94. The variables, namely, type of primary care facilities (*b* = −4.10; 95% CI: −5.80, −2.40; *P* < 0.001) and number of postnatal visits (*b* = 18.92; 95% CI: 18.37, 19.47; *P* < 0.001) added statistically significance to the estimation. However, education level (*b* = −2.66; 95% CI: −7.16, 1.84; *P* = 0.246) was not significant in the regression model for the estimation of total PNC cost.

### Postnatal Care Cost

The PNC cost by cost categories is shown in Table 6, where each input was expressed as a monetary value and as a percentage of the total. The mean PNC cost per patient in Negeri Sembilan for the year 2016 was RM165.65 (SD = 78.39). Personnel cost accounted for the highest proportion of the total cost at 94.2%, thus, contributing as the main cost driver for PNC (Table 5). Costs of investigation, drugs and others represented 1.7%, 1.4% and 2.7% of the total PNC cost, respectively. Other costs included all costs related to consumables and equipment used during the postnatal visit. The sensitivity analysis to evaluate the effect of variation in input costs of PNC cost in 2016 at public primary care showed that the average PNC cost was most sensitive to personnel cost.

Figure 1 illustrates a box plot of the PNC cost across the type of selected public primary care facilities in Negeri Sembilan. The plot showed that the facilities located in rural areas in Negeri Sembilan (Types 3, 5 and 6) had a higher medium cost of PNC (RM201.05–RM272.20) as compared to the cost attribute from the facilities in urban and semi-urban areas of Negeri Sembilan (Types 1, 2 and 4), with a median PNC cost of RM155.22–RM170.61.

### Total Postnatal Care Cost by Type of Pregnancy-Related Medical Conditions

As shown in Table 7, more than half (59.58%) of the women had at least one specified pregnancy-related problem. The common observed condition was anaemia (62.3%), followed by multiple complications (19.4%), diabetes (16.5%) and hypertension (1.8%). The mean PNC cost due to anaemia, diabetes, hypertension and multiple complications were RM163.21 (SD = 71.54), RM160.76 (SD = 81.72), RM148.54 (SD = 142.30) and RM172.37 (SD = 83.26) per person representing 35.4%, 9.5%, 0.9% and 12.3% of the total cost, respectively (Figure 2).

## Discussion

This pilot study assessed the cost of PNC per patient for the year 2016 in primary care facilities in Negeri Sembilan from the perspective of health providers. From the study findings, the average cost of PNC was RM165.65 per person per visit and personnel cost was found to be the PNC cost driver. This finding is in good agreement with previous studies reported that personnel cost often result as the highest cost in primary health care (20, 21). In Ethiopia, a study reported that medical supplies and personnel costs contributed the most to maternal and child health (14). However, a study by Zeng et al. (15) reported that the PNC cost estimated in an NGO-managed clinic in Bangladesh noted medicines as the primary PNC cost driver.

Given that the PNC service provided by health facilities in Malaysia is free of charge, this perhaps not contributes as the barrier for not seeking PNC at health facilities. Besides, studies reported that PNC utilisation was affected by several factors such as educational level, occupational status, maternal age, mode of delivery, place of delivery, number of pregnancies and awareness about PNC services (22–24). However, the exact findings could not be applied across different cultures and socioeconomic statuses within a society. In this study, it is interesting to note that the difference in PNC cost was affected by education level. Perhaps, this is similar to previous studies reported that education level plays an essential role in the utilisation of maternal health care (24–26). This probably could explain that the education level among mothers could improve health-seeking behaviour (27). Thus, it is understood that education level may influence the use of maternal health services.

There was a significant variation in the numbers of women visiting the health facilities between rural areas and urban and semi-urban areas. It is also notable that the PNC cost were significantly higher in rural areas compared to urban areas. Although facilities in rural areas received fewer PNC visitors, they presented higher PNC cost per person (RM205.61–RM271.33). This suggests an economies of scale, that is, if more mothers are mobilised to attend the healthcare facilities, the unit cost may be reduced (28). However, it is worth noting that this association may not present as a general trend to other health facilities or populations involved in such a study.

It was observed in this study that more than half of pregnancies were associated with at least one complication; in particular, anaemia was present in most complicated pregnancies. Likewise, anaemia is one of the most prevalent complications during pregnancy globally. It had been reported that the prevalence of anaemia in pregnant women is 38% and is less prevalent in developed countries at 9% than in developing countries at 43% (29–31). Although pregnancy and delivery are frequently compounded by complications that could lead to increased costs (31, 32), however, this is not the case for the present study.

This study comes with several limitations. To the best of the authors knowledge, no similar study such as this present one has been carried out to date. Therefore, the comparison of this the PNC cost from this study against other published studies will be complicated by the fact that other studies had reported on the antenatal care and total maternal care costs from a societal perspective. It can thus be suggested that such a study on PNC in particular in the future need to adopt a societal perspective and make use of a reference study to enable better comparisons across jurisdictions (33). In retrospect, this study employed a small-scale pilot study involving six public primary care facilities in Negeri Sembilan and one particular year of cost data. As a result, data from 2016 may not reflect the current postnatal cost. However, given this is a pilot study conducted in Negeri Sembilan, the different types of primary care we examined are geographically dispersed. It is acknowledged that the variation of primary care facilities across Malaysia in terms of resources available, utilisation and coverage of services, as well as types of service provided may differ. These suggest that results from this study could not be generalised to a national level. A more extensive data set involving health facilities from different states in Malaysia would provide more representative results.

In addition, the main challenge in this study relates to the availability of data from the record-keeping and health information systems at the primary care facilities. This study only focuses on the perspective of health providers, in which only the costs borne by the selected primary care facilities were taken into consideration. In other words, the cost borne by the patients/respondents were not included. Perhaps, a prospective cross-sectional study should be conducted to estimate the PNC cost from a social perspective. It is also acknowledged that the analysed cost data with a wide confidence interval was statistically significant, which ultimately left us uncertain about the magnitude of the association effect. Despite these limitations, the methodology employed in this study remains applicable across various settings.

## Conclusion

This study provided preliminary evidence from a small-scale sample analysis on the PNC cost from six public primary care facilities in Negeri Sembilan. The findings of this study revealed the cost of PNC per person per visit to be RM165.65 and personnel cost as the PNC cost driver. This study adds valuable insights to the evidence base of PNC cost and could serve as a reference for improving future estimates. The improved data will be of enormous use to the health facility managers and policymakers in instituting policy and controlling the healthcare budget allocation to ensure smooth delivery of maternal services in the country. Going forward, it remains a priority to provide more valuable cost data through the expansion of future studies, especially studies that involve larger datasets from health facilities across all states of Malaysia.

## Figures and Tables

**Figure 1:** Average PNC cost based on the type of selected public primary facilities in Negeri Sembilan

**Figure 2:** Pregnancy-related medical conditions cost breakdown

**Table 1:** Characteristics of public primary care facilities in Malaysia

Primary care facility	Catchment population	Building capacity (m^2^)	Daily patient attendance
Type 1	> 50,000	4,000	> 800
Type 2	> 50,000	4,000	500–800
Type 3	> 30,000–50,000	3,200	300–500
Type 4	> 20,000–30,000	2,500	150–300
Type 5	> 10,000–20,000	1,600	100–150
Type 6	> 5,000–10,000	700–800	50–100

Source: Ministry of Health Malaysia (18)

**Table 2:** Details of recurrent costs in the unit cost estimates

Recurrent Costs	Descriptions
**Personnel**	Comprised of basic salary and allowances of each staff involved in PNC. It was calculated as the FTE using time allocated by the staff to deliver postnatal-related work at the health facility.
**Facility utilities**	Comprised of electricity, water, telephone, internet, cleaning and waste management bills from the finance department of each health facility. The total expenditure was calculated using the ratio of maternal and child health department’s floor space over the total built-up area of the health facility, multiply by the number of patient.
**Laboratory tests**	The total number of laboratory investigations were multiplied by the reference costs.
**Consumables**	Comprised of the disposable items (gloves, surgical masks, injectable and cotton) that have been used during the service. The unit price of the consumables was calculated based on the purchase price provided by each health facility.
**Drugs**	The unit price of the drug was calculated from each medicine prescribed and written in the maternity book. The reference costs for medicine were based on the price list provided by the pharmacy department of each health facility.

**Table 3:** A mixed step-down and ABC approach

	Costing method	Unit measurement	Allocation factor
Capital cost			
Equipment	Step-down		PNC patient
Recurrent cost			
Personnel			
i. Administrative	Step-down		FTE
ii. Medical, pharmacy and lab	ABC	Minute	FTE
Utilities	Step-down		Floor space
Drugs	ABC	Minute	PNC patient
Laboratory tests	ABC	Minute	PNC patient
Consumables	ABC	Unit used	PNC patient

Notes: ABC = activity-based costing; FTE = full-time equivalent; PNC = postnatal care

**Table 4:** Sociodemographic characteristics and degree of variability by mean PNC

Variables	*n* (%)	mean (SD), RM	*F*-test	*P-*value	*t-*test
Age (years old)					
mean (SD): 29.59 (5.91)	287		0.38	0.541^b^	
< 20	11(3.8)	186.80 (63.07)			
20–29	131(45.7)	162.44 (82.99)			
30–39	134(46.7)	164.80 (74.01)			
> 40	11(3.8)	193.30 (88.93)			
Ethnicity			0.18	0.905^b^	
Malay	184 (64.1)	164.20 (84.74)			
Chinese	30 (10.5)	161.71 (75.02)			
Indian	55 (19.2)	169.33 (58.56)			
Others	18 (6.3)	175.91 (73.43)			
Marital status			1.55	0.435^a^	0.78
Married	274 (95.5)	164.87 (79.20)			
Not married	13 (4.5)	182.26 (58.53)			
Education level			2.90	**0.022** b	
Primary school	14 (4.9)	187.78 (100.39)			
Secondary school	144 (50.2)	177.96 (71.16)			
Certificate/ Diploma	75 (26.1)	155.80 (79.27)			
Bachelor’s degree	49 (17.1)	140.09 (86.99)			
Master’s/PhD	5 (1.7)	147.82 (33.99)			
Employment status			1.37	0.254^b^	
Housewife	126 (43.9)	171.26 (78.82)			
Student	4 (1.4)	210.01 (91.41)			
Non-professional	104 (36.2)	165.22 (73.56)			
Professional	53 (18.5)	149.86 (84.73)			
Current pregnancy-related illness			2.87	0.746^a^	0.41
Normal	119 (41.5)	167.45 (81.40)			
Complicated	168 (58.5)	164.39 (76.41)			
Type of primary care facility			16.82	< 0.01^b^	
Type 1	39 (14)	157.55 (73.57)			
Type 2	73 (25)	145.36 (64.30)			
Type 3	43 (15)	227.49 (98.86)			
Type 4	98 (34)	137.65 (55.09)			
Type 5	26 (9)	205.61 (44.28)			
Type 6	8 (3)	271.33 (116.77)			
Postnatal visit: mean (SD)	8.8 (4.07)				

Notes:

a Student’s *t*-test and

b one-way ANOVA tests were used for the analysis; *P* < 0.05 was considered statistically significant (*)

**Table 5:** Linear regression analysis of factors associated with total PNC cost

Variables	Simple linear regression		

	Unstandardised B coefficient	*P*-value	95% CI
Age	0.506	0.612	(−1.12, 2.13)
Ethnicity			
Malay	*Ref*		
Chinese	−2.487	0.873	(−32.99, 28.03)
Indian	5.125	0.672	(−18.69, 28.94)
Others	11.706	0.548	(−26.56, 49.98)
Marital status			
Married	*Ref*		
Not married	17.395	0.435	(−26.43, 61.22)
Education level			
Primary school	Ref		
Secondary school	24.209	0.009*	(6.179, 42.238)
Certificate/Diploma	–	–	–
Bachelor Degree	−2.031	0.734	(−62.25, 58.19)
Master/PhD	−17.743	0.132	(−79.31, 43.82)
Employment status			
Housewife	*Ref*		
Student	38.758	0.330	(−39.46, 116.97)
Non-professional	−6.041	0.560	(−26.44, 14.36)
Professional	−21.395	0.096	(−46.61, 3.82)
Current pregnancy-related illness			
Normal	*Ref*		
Complicated	−6.849	0.466	(−25.33, 11.63)
Type of health facilities			
Type 1	*Ref*		
Type 2	−12.186	0.377	(−39.28, 14.90)
Type 3	69.938	< 0.001**	(39.74, 100.14)
Type 4	−19.902	0.131	(−45.76, 5.96)
Type 5	48.059	0.007*	(13.48, 82.64)
Type 6	113.78	< 0.000**	(60.78, 166.79)
Postnatal visit	18.642	0.001**	(18.08, 19.20)

Notes: *Ref* = reference category; statistically significant at *P* < 0.05 (*) and *P* < 0.001 (**)

**Table 6:** PNC cost by cost categories

Cost category	PNC costs (RM)		

	Median (IQR), RM	Mean (SD), RM	%
Personnel	160.30 (76.58)	156.09 (75.24)	94.2
Investigation	4.42 (4.42)	2.83 (2.30)	1.7
Drug	0 (3.40)	2.28 (4.64)	1.4
Other	2.59 (3.41)	4.45 (5.32)	2.7

Total	167.12 (84.22)	165.65 (78.39)	100.0

Notes: Other costs include all consumables and equipment related to postnatal visit

**Table 7:** Cost by pregnancy-related medical conditions

Pregnancy-related medical conditions	*n* (%)	Average visits, *n* (days)	Total cost (RM)	

			Median (IQR), RM	Mean (SD), RM
Normal	119 (41.5)	8.6	172.34 (89.74)	167.45 (81.40)
Anaemia	103 (35.9)	8.8	166.56 (52.21)	163.21 (71.54)
Diabetes	28 (9.8)	8.4	162.76 (107.35)	160.76 (81.72)
Hypertension	3 (1.0)	7.7	126.96 (141.07)	148.54 (142.30)
Multiple	34 (11.8)	9.6	172.34 (82.13)	172.37 (83.26)

Total	287 (100.0)	8.8	167.12 (84.22)	165.65 (78.39)
